The article "Preoperative Body Composition Combined with Tumor Metabolism Analysis by PET/CT Is Associated with Disease-Free Survival in Patients with NSCLC" was published in 2022. Journal: Contrast Media Mol Imaging.

# Preoperative Body Composition Combined with Tumor Metabolism Analysis by PET/CT Is Associated with Disease-Free Survival in Patients with NSCLC

**DOI:** 10.1155/2022/7429319

**Published:** 2022-07-13

**Authors:** Hongpei Tan, Mengtian Ma, Jing Huang, Yuqian Dong, Jiahao Liu, Ze Mi, Kai Zheng, Shuo Hu, Pengfei Rong

**Affiliations:** ^1^Department of Radiology, Third Xiangya Hospital, Central South University, Changsha, China; ^2^Department of Anesthesiology, Zhuzhou Central Hospital, Zhuzhou, China; ^3^Department of Nuclear Medicine, Xiangya Hospital, Central South University, Changsha, China; ^4^PET/CT Center, Hunan Cancer Hospital, Changsha, China

## Abstract

**Objective:**

To evaluate the relationship between preoperative primary tumor metabolism and body composition in patients with NSCLC and analyze their effects on DFS.

**Method:**

A retrospective study was conducted on 154 patients with NSCLC. All patients were scanned by baseline 18F-FDG PET/CT. SUVmax (maximum standard uptake value) of primary tumor, liver SUVmean (mean standard uptake value), and spleen SUVmean were measured by AW workstation. The skeletal muscle area (SMA), skeletal muscle mass index (SMI), skeletal muscle radiation density (SMD), visceral fat area (VFA), visceral adipose tissue index (VATI), and skeletal muscle visceral fat ratio (SVR) were measured by ImageJ software. Kaplan–Meier survival analysis was used to evaluate the impact of the above parameters on DFS.

**Results:**

Compared with the low SUVmax group of primary tumors, the mean values of SMA, VFA, and VATI in the high SUVmax group were significantly higher. In addition, there were obvious differences in histopathological type, pathological differentiation, AJCC stage, and T stage between the two groups. Univariate analysis of DFS showed that VFA, VATI, pathological differentiation, tumor SUVmax, AJCC stage, tumor T stage, and N stage all affected the DFS of patients except for the parameters reflecting skeletal muscle content. Multivariate regression analysis showed that only VFA and SUVmax were associated with DFS. Kaplan–Meier survival analysis showed that high SUVmax, low VFA, high T stage, and high N stage were related to the decrease of DFS.

**Conclusion:**

：Preoperative ^18^F-FDG PET/CT could comprehensively evaluate the primary tumor SUVmax, skeletal muscle, and visceral fat in patients with NSCLC. The combination of primary tumor SUVmax and visceral fat area can well evaluate the prognosis of patients with NSCLC.

## 1. Introduction

Lung cancer is the leading cause of cancer deaths worldwide, accounting for 1/4 of all cancer deaths [1]. Surgical treatment is generally chosen for patients with non-small-cell lung cancer who have a chance of operation, but the prognosis of many patients is also very different, which may be related to the heterogeneity of the tumor itself or the condition of patients [2]. The body composition of the patients with myasthenia and fat thickness plays an important role in influencing the prognosis of lung cancer [3]. Body composition parameters obtained by CT scans have also been shown to be associated with prognosis in other tumors [4, 5]. Besides, 18F-FDG PET/CT has shown its ability to predict prognosis in many tumors [6, 7]. However, most studies only include the metabolic indicators of tumors without combining with body composition for analysis, in which CT parameters are mainly used for accurate histological localization. The CT scan in PET/CT can accurately quantify fat and muscle tissue and the standard examination of 18F-FDG PET/CT will cover the abdomen, so 18F-FDG PET/CT can be used to initially evaluate the body composition of the patients [8]. The purpose of this study was to evaluate the relationship between preoperative tumor metabolism and body composition and analyze their effects on disease-free survival in patients with non-small-cell lung cancer.

The article "Preoperative Body Composition Combined with Tumor Metabolism Analysis by PET/CT Is Associated with Disease-Free Survival in Patients with NSCLC" was published in 2022. Journal: Contrast Media Mol Imaging.

## 2. Methods

### 2.1. Patients

In this retrospective single-center study, patients were selected from the institutional database using the following inclusion/exclusion criteria. Inclusion criteria were as follows: (a) older than 18 years old, less than 90 years old; (B) patients who underwent surgical resection of cancer lesions in lung between 2008 and 2015; (c) fluoro-18 fluorodeoxyglucose positron emission tomography/computed tomography (^18^FFDG PET/CT) scan was performed in our facility 45 days before operation to identify lung lesions. Exclusion criteria were as follows: (a) nonlung adenocarcinoma or squamous cell carcinoma; (B) associated with other cancer types or previous cancers; (C) distant metastases; (D) no PET/CT whole-body scan; (E) patients with tumors larger than 7 cm; (F) patients with other diseases, such as cardiovascular disease, diabetes, or liver or spleen disease; and (F) incomplete follow-up information. A total of 154 patients were selected for the study according to the above inclusion and exclusion criteria.

In this study, DFS was used as the standard to evaluate the prognosis. DFS is defined as the time between the date of operation and the date of recurrence (event), which is referred to the date of tumor recurrence, tumor-related death, or the date of the last visit (after examination). The follow-up interval of patients was 6 months in the first three years, and then once a year. All patients were followed up for at least 5 years, recurrence or death within 5 years was defined as the occurrence of an event, and the last follow-up was in 2021. This study was approved by the Institutional Ethics Committee.

The article "Preoperative Body Composition Combined with Tumor Metabolism Analysis by PET/CT Is Associated with Disease-Free Survival in Patients with NSCLC" was published in 2022. Journal: Contrast Media Mol Imaging.

### 2.2. PET/CT Examination

18F-FDG PET/CT image acquisition was carried out according to version 1.0 of the European Association of Nuclear Medicine (EANM) guidelines by an integrated PET/CT scanner (General Electric Healthcare, Chicago, IL). Images were obtained 60 ± 5 minutes after the intravenous injection of 18F-FDG at a dose of 370 MBq/kg. Firstly, a low-dose CT scan without contrast enhancement (120 mA, 150 kV, 512 × 512 matrix, the pitch of 1.75, reconstruction thickness, and interval of 3.75 mm) was performed for a precise anatomical localization and attenuation correction. Next, a three-dimensional PET scan (thickness of 3.27 mm) was performed from the skull base to the proximal thighs with an acquisition time of 3 min per bed position. The PET data sets were iteratively reconstructed using an ordered-subset expectation maximization (OSEM) algorithm with attenuation correction. All collected images were displayed on the GE Healthcare Xeleris 3.0 to reconstruct the fusion images.

### 2.3. PET/CT Image Analysis

Two senior nuclear medicine doctors who did not know the clinical information of the patients evaluated PET/CT images, respectively, both of them had more than 5 years of experiences in PET/CT diagnosis. The size of the tumor was determined on the maximum cross-sectional plane, which was depicted around the tumor outline on CT and PET images. The ROI was carefully placed on different cross sections of the primary tumor to measure the maximum standardized uptake of the primary tumor (SUVmax). Some studies have shown that tumors affect the metabolism of distal organs, so we also included the metabolism of the liver and spleen in this study [9, 10]. We select a more uniform region in the liver parenchyma of the largest cross section of the liver right lobe and draw a circle with a diameter not less than 3 cm as ROI. The liver SUVmean of each patient was measured three times, and the average value was calculated to reduce the selection deviation [7]. Similarly, the largest cross section of the spleen was selected and the ROI was drawn in a relatively uniform parenchyma. The spleen SUVmean was the average value of three times measurement in each patient [11]. Tumor size is defined as the maximum diameter of the primary tumor. Regional lymph nodes and distant metastases were evaluated according to the eighth edition of the AJCC staging system.

### 2.4. Quantification of Body Composition

The relevant body components were measured in the baseline CT images of the third vertebral body level (L3) obtained from patients. Each selected CT image is evaluated by two reviewers who do not know the end point. A free program was used in this study, which has been previously verified to provide reliable measurement results (NIH ImageJ version 1.53c, https://imagej.nih.gov/ij/) [12, 13]. Skeletal muscle area (SMA, cm^2^) used a standard threshold of +29 ∼ +150 Hounsfield units (HU) to measure. Skeletal muscle mass index (SMI, cm^2^/m^2^) obtained by dividing the area of skeletal muscle by the square of height. Radiation density of skeletal muscle (SMD, HU) draws the ROI in the relevant skeletal muscle area for measurement. Visceral fat area (VFA, cm^2^) used a standard threshold of −150∼−50 HU to measure. Visceral adipose tissue index (VATI, cm^2^/m^2^) divided the visceral fat area by the square of height. Using SMA divided by VFA to obtain skeletal muscle and visceral fat ratio (SVR). Based on the previously established gender-specific threshold from healthy adults, low SMI or myopenia is defined as SMI <44.4 cm^2^/m^2^ in male and <34.8 cm^2^/m^2^ in female, and low SMD or myosteatosis is defined as SMD <34.1 HU in male and <27.2 HU in female. Sarcopenia is defined as the presence of myopenia or myoosteogenesis according to the operational definition of sarcopenia recommended by EWGSOP2 [14]. According to the obesity standard of Japan Obesity Research Association, VFA is divided into H-VFA (≥100 cm^2^) and L-VFA (<100 cm^2^) [15].

The article "Preoperative Body Composition Combined with Tumor Metabolism Analysis by PET/CT Is Associated with Disease-Free Survival in Patients with NSCLC" was published in 2022. Journal: Contrast Media Mol Imaging.

### 2.5. Statistical Analysis

Student's *t* test or Mann–Whitney *U* test was used to estimate the differences between groups according to the normal distribution. Chi-squared test or Fisher's exact test was used to estimate the differences between groups for categorical data. Cumulative survival was plotted using the Kaplan–Meier method, and differences were compared using the log-rank test. Cox proportional-hazards model was used for univariate and multivariate analyses of potential risk factors. Hazard ratios (HRs) together with 95% confidence intervals (CI) were provided. All statistical analyses were performed with the R software, version 4.12 (http://www.r-project.org).

## 3. Results

### 3.1. Basic Characteristics of Patients

The baseline characteristics of the patients are shown in Table 1. A total of 154 patients were included in the study, which included 46 women and 108 men, with an average age of 58 years. The average SUVmax of primary tumor was 8.41. The patients with moderately differentiated tumor account large percentage. The proportion of patients in low level of staging is larger than that of patients in other stages according to the AJCC staging (Table 1).

The article "Preoperative Body Composition Combined with Tumor Metabolism Analysis by PET/CT Is Associated with Disease-Free Survival in Patients with NSCLC" was published in 2022. Journal: Contrast Media Mol Imaging.

### 3.2. Correlation between Tumor Metabolism, Body Composition, and Clinical Parameters

We divided the patients into groups according to the level of SUVmax. Patients with higher SUVmax had higher BMI index, skeletal muscle area, and visceral fat area, as well as less differentiated tumors and a higher proportion of squamous cell carcinoma, while their tumors are larger and their AJCC stages are higher (Table 2).

### 3.3. Univariate and Multivariate Analysis of Disease-Free Survival

We evaluated the effect of various indicators on postoperative disease-free survival of patients，Univariate analysis showed that visceral fat area (HR: 0.99, 95%CI, 0.98–0.99, *P* < 0.001), visceral fat index (HR: 0.97, 95%CI, 0.96–0.98, *P* < 0.001), pathological differentiation (HR: 0.68, 95%CI, 0.49–0.96, *P* < 0.05), and SUVmax (HR: 1.1, 95%CI, 1.1–1.2, *P* < 0.001)，AJCC stage (HR: 1.7, 95%CI, 1.3–2.3, *P* < 0.001), T stage (HR: 1.6, 95%CI, 1.2–2, *P* < 0.001), and lymph node staging (HR: 1.6, 95%CI, 1.2–2.1, *P* < 0.01) can affect the disease-free survival of patients. Multivariate regression analysis showed that only visceral fat area (HR: 0.98, 95%CI, 0.97–1.00, *P* < 0.05) and SUVmax (HR: 1.14, 95%CI, 1.08–1.20, *P* < 0.001) were associated with disease-free survival (Figure 1).

### 3.4. Kaplan–Meier Survival Analysis

Kaplan–Meier survival analysis showed that high SUVmax, low VFA, high T stage, and high N stage were related to the decrease of disease-free survival (Figure 2). It was found that tumor SUVmax combined with VFA could better predict the DFS of patients by comparing the survival curve generated by the combination of tumor SUVmax, VFA, and AJCC staging, which showed that the patients with low tumor SUVmax and H-VFA had better DFS (Figure 3).

## 4. Discussion

Body composition and tumor glucose metabolism are known as prognostic markers for cancer patients. Our study shows the prognostic value of preoperative PET/CT analysis of body composition and tumor glucose metabolism for disease-free survival in patients with non-small-cell lung cancer. In our study, tumor SUVmax, visceral fat area, visceral fat index, tumor differentiation, and various clinical stages were all risk factors for disease-free survival. Combining visceral fat area and tumor SUVmax can better determine the risk of disease-free survival compared with AJCC stage, while there is no relationship between the indexes of muscle and disease-free survival.

Glucose metabolism is very important for tumor growth and development. 18F-FDG PET/CT is often used for preoperative evaluation and grading of patients with lung cancer [16], SUVmax is a commonly used parameter to measure tumor metabolism in clinic [17]. Our results show patients with higher SUVmax have higher BMI index, skeletal muscle area, and visceral fat area, as well as less differentiated tumors and a higher proportion of squamous cell carcinoma, while their tumors are larger and their AJCC stages are higher. These results may also be the reason for the shorter disease-free survival time of patients with high SUVmax.

The article "Preoperative Body Composition Combined with Tumor Metabolism Analysis by PET/CT Is Associated with Disease-Free Survival in Patients with NSCLC" was published in 2022. Journal: Contrast Media Mol Imaging.

Every year, nearly 500000 of new cancers are caused by obesity. Avoiding obesity can reduce the incidence of cancer. This conclusion has been strongly supported by data in a variety of tumors [18]. However, in some tumors, there is no significant correlation between higher BMI and mortality in diagnosed patients, a phenomenon also known as fat paradox [19–21], A summary study found that there was no significant difference in mortality between tumor patients with BMI ≥ 25 kg/m^2^ and those with BMI ≤ 18 < 25 kg/m^2^ [22]. In fact, many studies have reported that patients with higher BMI have obvious survival advantages, including lymphoma, gastric cancer, colorectal cancer, and lung cancer [23–26]. One possible explanation is that BMI cannot reflect the content and proportion of individual muscle and fat, so it cannot fully reflect the patient's physical condition, thus negatively affecting the correlation between obesity degree and clinical outcome. As an important way of energy storage, fat plays an important role in many aspects, such as metabolism and immunity [12, 27]. In tumor patients, fat consumption generally precedes muscle atrophy, so the decrease of survival time caused by fat deficiency may be related to the decrease of energy reserves and the destruction of energy balance in cancer patients [28, 29]. In this study, our results show that high visceral fat area is beneficial for disease-free survival in patients with NSCLC, but the role of visceral fat in NSCLC may be multifaceted, and it has shown that visceral fat index can affect OS and RFS in patients with NSCLC and inhibit immune response [30]; however, there are also studies showing that although visceral fat is associated with tumor progression and immune disorders, it is also associated with immune cell infiltration in the tumor area, making it easier to benefit from immunotherapy and achieve better OS [31, 32]. A recent study shows that the visceral fat area and inflammation-related indexes of NSCLC patients treated with pembrolizumab are significantly increased during treatment [33], and studies have confirmed that obese NSCLC patients are more likely to benefit from immunotherapy [34, 35], so visceral fat may play an important role in immune regulation. At the same time, some studies have also shown the impact of VFA on the prognosis of other tumors [36, 37]. Therefore, VFA is worthy of attention in tumor research. Studies have shown that sarcopenia is associated with shorter OS in lung cancer patients, but does not appear to influence DFS [38], which is consistent with our results that muscle index and sarcopenia have no significant effect on disease-free survival. However, more multicenter studies may be needed to confirm this conclusion.

The article "Preoperative Body Composition Combined with Tumor Metabolism Analysis by PET/CT Is Associated with Disease-Free Survival in Patients with NSCLC" was published in 2022. Journal: Contrast Media Mol Imaging.

PET/CT is recommended to determine the stage of disease in patients with lung cancer before treatment and abdominal and L3 levels are generally selected for the evaluation of fat and muscle, so the results of a whole-body PET/CT scan can make a comprehensive analysis of the patient's body composition and body metabolism without the need for additional examination. Our results also show that the combination of tumor metabolism and visceral fat area can better evaluate the prognosis of patients. We do not distinguish brown adipose tissue in the quantitative evaluation of fat, which may be helpful to study the effect of fat on patients' survival according to some studies, showing that brown adipose tissue plays an important role in tumors [13, 39].

Our study still has some limitations. First of all, our study is a single-center retrospective study with limited sample size, and further multicenter studies are needed to verify our conclusions. In addition, we only studied the effects of body composition combined with tumor glucose metabolism on disease-free survival, and it may be more meaningful when combined with the overall survival.

## 5. Conclusion

Our study shows that preoperative PET/CT could comprehensively evaluate the metabolic level and body composition of patients with non-small-cell lung cancer, and the combination of tumor glucose metabolism and visceral fat area can better predict the prognosis of patients.

## Figures and Tables

**Figure 1:** Univariate (a) and multivariate (b) Cox regression analysis of clinical indicators, metabolic, and body composition parameters.

**Figure 2:** Kaplan–Meier survival analysis curves showing differences in disease-free survival across different subgroups in NSCLC. VFA (a), SUVmax (b), T stage (c), and N stage (d).

**Figure 3:** Kaplan–Meier survival curve of VFA combined with SUVmax (a); Kaplan–Meier survival curve of AJCC clinical stages (b).

**Table 1:** Baseline characteristics of patients.

Characteristic (mean ± SD)	All patients (*n* = 154)
Gender (%)	
Female	46 (29.9)
Male	108 (70.1)
Age	58.49 (9.39)
BMI	22.85 (3.47)
SMA	110.71 (21.88)
SMI	43.82 (4.15)
SMD	44.00 (3.24)
VFA	115.70 (56.52)
VATI	43.26 (20.74)
SVR	1.19 (0.59)
Sarcopenia (%)	
Without	74 (48.1)
With	80 (51.9)
Pathology (%)	
Adenocarcinoma	88 (57.1)
Squamous carcinoma	66 (42.9)
Differentiation (%)	
Poor	50 (32.5)
Moderate	73 (47.4)
Well	31 (20.1)
SUVmax	8.41 (4.55)
Liver SUVmean	2.16 (0.43)
Spleen SUVmean	1.84 (0.35)
AJCC stage	
Stage I	73 (47.4)
Stage II	46 (29.9)
Stage III	35 (22.7)
T stage (%)	
T1	68 (44.2)
T2	61 (39.6)
T3	16 (10.4)
T4	9 (5.8)
N stage (%)	
N0	104 (67.5)
N1	24 (15.6)
N2	26 (16.9)

SUVmax, maximum standard uptake value; SUVmean, mean standard uptake value; BMI, body mass index; SMA, skeletal muscle area; SMI, skeletal muscle mass index; SMD, skeletal muscle radiation density; VFA, visceral fat area; VATI, visceral adipose tissue index; SVR, skeletal muscle visceral fat ratio.

The article "Preoperative Body Composition Combined with Tumor Metabolism Analysis by PET/CT Is Associated with Disease-Free Survival in Patients with NSCLC" was published in 2022. Journal: Contrast Media Mol Imaging.

**Table 2:** Relationship between primary tumor SUVmax, body composition, and clinical features.

Characteristic (mean ± SD)	SUVmax		
	Low (*n* = 77)	High (*n* = 77)	*P*
Gender (%)			0.379
Female	26 (33.8)	20 (26.0)	
Male	51 (66.2)	57 (74.0)	
Age^†^	60.00 [53.00, 66.00]	59.00 [51.00, 64.00]	0.253
BMI^†^	21.78 [19.78, 24.17]	23.19 [21.10, 25.34]	0.015
SMA (cm^2^)	106.35 (21.00)	115.08 (22.01)	0.013
SMI	43.61 (3.94)	44.03 (4.36)	0.533
SMD (HU)	43.68 (3.08)	44.33 (3.38)	0.212
VFA^†^ (cm^2^)	92.86 [61.96, 137.17]	123.08 [72.69, 166.21]	0.005
VATI^†^	34.48 [23.28, 53.16]	45.40 [28.42, 61.33]	0.017
SVR^†^	1.10 [0.78, 1.60]	0.90 [0.70, 1.38]	0.065
Sarcopenia (%)			0.872
Without	38 (49.4)	36 (46.8)	
With	39 (50.6)	41 (53.2)	
Pathology (%)			0.002
Adenocarcinoma	54 (70.1)	34 (44.2)	
Squamous carcinoma	23 (29.9)	43 (55.8)	
Differentiation (%)			<0.001
Poor	19 (24.7)	31 (40.3)	
Moderate	33 (42.9)	40 (51.9)	
Well	25 (32.5)	6 (7.8)	
SUVmax^†^	—	—	
Liver SUVmean^†^	2.09 [1.87, 2.46]	2.25 [2.01, 2.49]	0.09
Spleen SUVmean^†^	1.84 [1.60, 2.03]	1.91 [1.72, 2.03]	0.208
AJCC stage			<0.001
Stage I	51 (66.2)	22 (28.6)	
Stage II	16 (20.8)	30 (39.0)	
Stage III	10 (13.0)	25 (32.5)	
T stage (%)			<0.001
T1	53 (68.8)	15 (19.5)	
T2	19 (24.7)	42 (54.5)	
T3	4 (5.2)	12 (15.6)	
T4	1 (1.3)	8 (10.4)	
N stage (%)			0.052
N0	59 (76.6)	45 (58.4)	
N1	9 (11.7)	15 (19.5)	
N2	9 (11.7)	17 (22.1)	

^†^Non-normal distribution, quartile.

## Data Availability

The data used to support the findings of this study are available from the corresponding author upon request.
